# LncRNA SRA1 is down-regulated in HPV-negative cervical squamous cell carcinoma and regulates cancer cell behaviors

This article has been retracted.

**DOI:** 10.1042/BSR20191226

**Published:** 2019-08-15

**Authors:** Yunyong Liu, Mengdan Li, Huihui Yu, Haozhe Piao

**Affiliations:** 1 Department of Cancer Prevention and Control, Cancer Hospital of China Medical University, Liaoning Cancer Hospital and Institute, Shenyang City 110042, Liaoning Province, P.R. China; 2 Department of Neurosurgery, Cancer Hospital of China Medical University, Liaoning Cancer Hospital and Institute, NO. 44 Xiaoheyan Road, Dadong District, Shenyang City 110042, Liaoning Province, P.R. China

**Keywords:** cervical squamous cell carcinoma, HPV, lncRNA SRA1, miR-9

## Abstract

LncRNA SRA1 plays important roles in several types of human diseases. The present study aimed to explore the role of SRA1 in cervical squamous cell carcinoma (CSCC). In the present study, we showed that plasma SRA1 was down-regulated in human papillomavirus (HPV)-negative CSCC patients but not in HPV-positive CSCC patients compared with healthy females. Down-regulated SRA1 distinguished HPV-negative CSCC patients from HPV-positive CSCC patients and healthy females. In HPV-negative CSCC patients, miR-9 was up-regulated and inversely correlated with SRA1. In HPV-negative CSCC cells, SRA1 overexpression caused the down-regulated miR-9, while miR-9 overexpression failed to affect SRA1. Moreover, SRA1 overexpression caused decreased, while miR-9 overexpression caused increased proliferation, migration and invasion rates of cancer cells. In addition, miR-9 overexpression attenuated the effects of SRA1 overexpression. Therefore, SRA1 is down-regulated in HPV-negative CSCC and regulates cancer cell behaviors possibly by down-regulating miR-9.

## Introduction

In both developing and developed countries, cervical cancer is a common female malignancy and causes unacceptable high mortality rate [1]. Due to the low early diagnostic rate, only a small portion of cervical cancer patients are candidates for radical surgery [2]. Most patients with cervical cancer are diagnosed at advanced stages and overall 5-year survival rate is generally below 20% [3]. Human papillomavirus (HPV) infection is the major cause of cervical cancer. The popularization of HPV vaccines and early screening program has significantly reduced the incidence rate of cervical cancer [4]. However, incidence of HPV-negative cervical cancer, which is a more malignant form of cervical cancer comparing with the HPV-positive subtype, showed an increasing trend in recent years [5,6].

Pathogenesis of HPV-negative cervical cancer has not been well studied. However, previous studies have revealed the different gene expression patterns of HPV-negative and HPV-positive subtypes of this disease [7,8], indicating that they have different molecular pathways involved. Long non-coding RNAs (lncRNAs, >200 nt) lack protein coding capacity but play pivotal roles in cancer biology by regulating gene expression [9]. A recent study reported an lncRNA named snaR is involved in the recurrence of HPV-negative but not HPV-positive cervical squamous cell carcinoma (CSCC, a major subtype of cervical cancer) [10], indicating the involvement of lncRNAs in HPV-negative CSCC. In a recent study, Lu et al. reported a novel lncRNA SRA1 as a potential tumor suppressive lncRNA in hepatocellular carcinoma [11]. Our preliminary transcriptome analysis data showed that SRA1 was down-regulated in HPV-negative but not in HPV-positive CSCC patients. This lncRNA attracted our attention and the present study was carried out to characterize the function of SRA1 in CSCC.

## Materials and methods

### Study patients

Our study selected 72 CSCC patients (35–67 years, 46.7 ± 5.2 years) from the 133 CSCC patients who were admitted to the Cancer Hospital of China Medical University, Liaoning Cancer Hospital and Institute between December 2015 and December 2018. Inclusion criteria: (i) new CSCC cases diagnosed by histopathological examinations and (ii) patients willing to join the study. Exclusion criteria: (i) recurrent CSCC; (ii) any therapies performed within 3 months before admission; (iii) family history of malignancies and (iv) previous history of malignancies. Sensitive PCR was performed to detect the HPV infections. The results revealed 16 HPV-11 positive cases, 20 HPV-16 positive cases, 14 HPV-18 positive cases and 22 HPV-negative cases. During the same time period, 72 healthy females (36–66 years, 47.1 ± 5.5 years) were also selected at the Physical Health Center of Cancer Hospital of China Medical University, Liaoning Cancer Hospital and Institute to serve as controls. These two groups of participants showed similar age distributions. Ethics Committee of the aforementioned hospital approved the present study.

### Plasma and cells

Fasting blood (5 ml) was extracted from each CSCC patient and healthy control on the day of admission before the initiation of any therapies. Blood was centrifuged in EDTA-treated tubes and was centrifuged at 1200×***g*** for 10 min to collect plasma.

### C33A HPV-negative CSCC cell line was used in the present study

HPV-negative human CSCC cell line C-33 A. Eagle’s Minimum Essential Medium containing 10% fetal bovine serum (FBS) was used as cell culture medium and cell culture conditions were 37°C and 5% CO_2_.

### RT-qPCR

TRIzol reagent (Invitrogen, U.S.A.) was mixed with plasma and C-33 A cells to extract total RNAs. Following DNase I digestion, RNA samples were subjected to reverse transcription using AMV Reverse Transcriptase (Canvax Biotech, U.S.A.) to synthesize cDNA. SYBR Green for qPCR (Bio-Rad, U.S.A.) was used to prepare PCR mixtures with 18S rRNA as endogenous control to detect the expression of SRA1.

MiRNAs were extracted from plasma and C-33 A cells using microRNA Purification Kit (Cat. 21300, Norgen Biotek Corp, U.S.A.). qScript microRNA cDNA Synthesis Kit (Quantabio, U.S.A.) was used to perform miRNA reverse transcriptions and miScript SYBR Green PCR Kit (QIAGEN, Germany) was used to prepare PCR with U6 as endogenous control to detect the expression of miR-9.

All PCR were repeated three times and all *C*_t_ values were processed using 2^−ΔΔ*C*^_T_ method.

### Vectors and transient cell transfections

SRA1 expression vector was constructed using pcDNA3.1 vector (Sangon, Shanghai, China). Negative control (NC) miRNA and miR-9 mimic were bought from Sigma–Aldrich (U.S.A.). C-33 A cells were collected when confluence reached 70–80%. Lipofectamine 2000 reagent (11668-019, Invitrogen, U.S.A.) was used to transfect 10 nM SRA1 expression vector, 10 nM empty pcDNA3.1 vector (NC), 30 nM miR-9 mimic or 30 nM NC miRNA (NC) into 10^5^ cells. Cells with no transfections were also included to serve as control group (C). Following studies were performed using cells harvested at 24 h after transfection.

### Measurement of cell proliferation abilities

C-33 A cells were harvested at 24 h after transfection, and 4 × 10^4^ cells were mixed with 1 ml Eagle’s Minimum Essential Medium containing (10%, FBS) to prepare single cell suspensions. A 96-well cell culture plate was used to cultivate the cells with 0.1 ml per well. Cells were cultivated under the conditions of 37°C and 5% CO_2._ CCK-8 solution (10 μl) was added 22, 46, 70 and 94 h later, and cells were harvested 24, 48, 72 and 96 h later. After that, DMSO (10 μl) was added into each well and OD values were measured at 450 nm to reflect cell proliferation.

### Measurement of cell migration and invasion abilities

C-33 A cells were harvested at 24 h after transfections, and 4 × 10^4^ cells were mixed with 1 ml non-serum Eagle’s Minimum Essential Medium to prepare single cell suspensions. The upper Transwell chamber was filled with 0.1 ml cell suspension and the lower chamber was added with Eagle’s Minimum Essential Medium containing 20% FBS. Matrigel (50 μl/filter; BD Biosciences, U.S.A.) was used to coat the upper chamber membrane before invasion assay to mimic *in vivo* invasion conditions. Transwell chambers were cultivated under conditions of 37°C and 5% CO_2_ for 4 h and staining with 0.5% Crystal Violet (Sigma–Aldrich; Merck KGaA) was performed for 20 min at 22°C. Stained cells were observed and counted under an optical microscope.

### Data analysis

Data presented in the present paper were mean values of three biological replicates. Differences among different groups of participants or among different cell transfection groups were analyzed using one-way ANOVA and Tukey’s test. Linear regression was used for correlation analysis. Diagnostic analyses were performed using ROC curve analysis. *P*<0.05 was statistically significant.

## Results

### SRA1 was down-regulated in HPV-negative CSCC patients

The 72 CSCC patients included 16 HPV-11 positive cases, 20 HPV-16 positive cases, 14 HPV-18 positive cases and 22 HPV-negative cases. SRA1 in plasma of all CSCC patients and healthy controls (*n*=72) was detected by performing RT-qPCR. Plasma levels of SRA1 among those groups of participants were compared by performing one-way ANOVA and Tukey’s test. Compared with Control group, significantly lower plasma levels of SRA1 were found in the 22 HPV-negative patients but not in other groups of patients (Figure 1, *P*<0.05).

**Figure 1:** SRA1 was down-regulated in HPV-negative CSCC patients Plasma levels of SRA1 compared by one-way ANOVA and Tukey’s test showed that, compared with Control group, significantly lower plasma levels of SRA1 were found in the 22 HPV negative patients but not in other groups of patients (*, *P*<0.05).

### Altered plasma levels of SRA1 showed diagnostic values for HPV-negative CSCC

Diagnostic values of plasma SRA1 for HPV-negative CSCC were analyzed by performing ROC curve analysis. With healthy controls as true negative cases, area under the curve (AUC) was 0.86, with standard error of 0.050 and 95% confidence interval of 0.76–0.96 (Figure 2A). With HPV-positive cases as true negative cases, AUC was 0.95, with standard error of 0.025 and 95% confidence interval of 0.90–0.99 (Figure 2B).

**Figure 2:** Altered plasma levels of SRA1 showed diagnostic values for HPV-negative CSCC Down-regulated SRA1 distinguished HPV-negative CSCC patients from healthy females (**A**) and HPV-positive CSCC patients (**B**).

### SRA1 down-regulated miR-9 in HPV-negative CSCC cells

MiR-9 in plasma of HPV-negative patients was detected by performing RT-qPCR. Correlation between miR-9 and SRA1 was analyzed by performing linear regression. It was observed that miR-9 and SRA1 were inversely and significantly correlated in HPV-negative CSCC patients (Figure 3A). To further analyze the relationship between miR-9 and SRA1, miR-9 mimic and SRA1 expression vector were transfected into cells of HPV-negative CSCC cell line C-33 A. Compared with C and NC groups, expression levels of miR-9 and SRA1 were significantly up-regulated at 24 h after transfections (Figure 3B, *P*<0.05). Moreover, SRA1 overexpression caused the down-regulated miR-9, while miR-9 overexpression failed to affect SRA1 expression (Figure 3C, *P*<0.05).

**Figure 3:** SRA1 down-regulated miR-9 in HPV-negative CSCC cells Linear regression revealed that miR-9 and SRA1 were inversely and significantly correlated in HPV-negative CSCC patients (**A**). Comparing with C and NC groups, expression levels of miR-9 and SRA1 were significantly up-regulated at 24 h after transfections (**B**). Moreover, SRA1 overexpression caused the down-regulated miR-9, while miR-9 overexpression failed to affect SRA1 expression (**C**) (*, *P*<0.05).

### SRA1 regulated HPV-negative CSCC cell behaviors through miR-9

Cell proliferation, migration and invasion abilities of C-33 A were tested 24 h after transfections. Comparing with C and NC groups, SRA1 overexpression caused decreased, while miR-9 overexpression caused increased proliferation (Figure 4A), migration (Figure 4B) and invasion (Figure 4C) rates of C-33 A cells (*P*<0.05). In addition, miR-9 overexpression attenuated the effects of SRA1 overexpression.

**Figure 4:** SRA1 regulated HPV-negative CSCC cell behaviors through miR-9 Cell proliferation, migration and invasion abilities of C-33 A were tested at 24 h after transfections by performing CCK-8 assay and Transwell migration and invasion assay, respectively. Comparing with C and NC groups, SRA1 overexpression caused decreased, while miR-9 overexpression caused increased proliferation (**A**) migration (**B**) and invasion (**C**) rates of C-33 A cells. In addition, miR-9 overexpression attenuated the effects of SRA1 overexpression (*, *P*<0.05).

### SRA1 and miR-9 regulated p53 but not E6, E7 and NF-κb in HPV-negative CSCC cells

The expression levels of E6 (Figure 5A), E7 (Figure 5B), NF-κb (Figure 5C) and p53 (Figure 5D) in C-33 A cells were measured at 24 h after transfection. Compared with C and NC groups, SRA1 and miR-9 overexpression failed to affect E6, E7 and NF-κb. However, SRA1 overexpression caused decreased, while miR-9 overexpression caused increased expression level of p53. In addition, miR-9 overexpression attenuated the effects of SRA1 overexpression (*P*<0.05).

**Figure 5:** SRA1 and miR-9 regulated p53 but not E6, E7 and NF-κb in HPV-negative CSCC cells The expression levels of E6 (**A**) E7 (**B**) NF-κb (**C**) and p53 (**D**) in C-33 A cells were measured at 24 h after transfections. Comparing with C and NC groups, SRA1 and miR-9 overexpression failed to affect E6, E7 and NF-κb. However, SRA1 overexpression caused decreased, while miR-9 overexpression caused increased expression level of p53. In addition, miR-9 overexpression attenuated the effects of SRA1 overexpression (*, *P*<0.05).

## Discussion

In the present study, we investigated the involvement of SRA1 in two types of CSCC. We found that SRA1 was only down-regulated in HPV-negative CSCC and overexpression of SRA1 caused the inhibited cancer cell behaviors. We also showed that the actions of SRA1 in HPV-negative CSCC are likely mediated by miR-9, which is up-regulated in CSCC [12].

Previous studies have identified a considerable number of differentially expressed lncRNAs in CSCC [13]. LncRNA GAS5 was down-regulated in CSCC and overexpression of GAS5 suppressed the development of CSCC by down-regulating two oncogenic miRNAs, miR-196a and miR-205 [14]. In contrast, lncRNA XIST was up-regulated in CSCC and promoted cancer progression [15]. Moreover, dysregulation of certain lncRNAs, such as MALAT1 and NCK1-AS1 also participate in the regulation of radiosensitivity and chemosensitivity of CSCC cells, thereby affecting treatment outcomes [16,17]. However, it is known that HPV-positive and -negative CSCC have different pathogenesis. Those studies failed to identify an lncRNA that can be used to distinguish those two subtypes. Our data showed that SRA1 was down-regulated only in HPV-negative CSCC and the down-regulation of SRA1 distinguished HPV-negative CSCC patients from HPV-positive CSCC patients and healthy controls. Our study further confirmed the different gene expression patterns involved in these two subtypes of CSCC and provide a potential diagnostic marker to distinguish these two subtypes.

Interestingly, our study showed that SRA1 down-regulated miR-9 to suppress HPV-negative CSCC cell proliferation, migration and invasion. It has been reported that miR-9 was up-regulated in both HPV-negative and -positive CSCC [12]. Therefore, HPV-negative and -positive CSCC may have different pathways on the upstream of miR-9, while both types require the involvement of up-regulation of miR-9. These data provided new insights to the pathogenesis of two subtypes of CSCC. In addition, overexpression of SRA1 may serve as potential therapeutic target for HPV-negative CSCC. However, more clinical studies are needed to further confirm our conclusions.

In addition, SRA1 was down-regulated specifically in HPV-negative CSCC. SRA1 may suppress HPV-negative CSCC behaviors by down-regulating miR-9.

E6 and E7 are critical players in HPV-associated cervical carcinogenesis [18]. Consistently, our study showed that SRA1 and miR-9 had no significant effects on E6 and E7 expression. Cancer development is closely correlated with inflammation, in which p53 and NF-Kb play pivotal roles [19–21]. It is also known that, non-coding RNAs, such as lncRNAs, are master regulators of inflammatory signaling [22]. In our study we showed that SRA1 and miR-9 can interact with each other to regulate p53. Therefore, a novel SRA1/miR-9/p53 pathway in HPV-negative CSCC was characterized.

## Availability of data and materials

The analyzed datasets generated during the study are available from the corresponding author on reasonable request.

## Abbreviations

AUC: area under the curve
CSCC: cervical squamous cell carcinoma
FBS: fetal bovine serum
HPV: human papillomavirus
lncRNA: long non-coding RNA
NC: negative control

## References

[1] JemalA., BrayF., CenterM.M., FerlayJ., WardE. and FormanD. (2011) Global cancer statistics. CA Cancer J. Clin.61, 69–9010.3322/caac.2010721296855

[2] DasariS., WudayagiriR. and ValluruL. (2015) Cervical cancer: biomarkers for diagnosis and treatment. Clin. Chim. Acta445, 7–1110.1016/j.cca.2015.03.00525773118

[3] Diaz-PadillaI., MonkB.J., MackayH.J. and OakninA. (2013) Treatment of metastatic cervical cancer: future directions involving targeted agents. Crit. Rev. Oncol. Hematol.85, 303–31410.1016/j.critrevonc.2012.07.00622883215

[4] ChabedaA., YanezR.J.R., LamprechtR. (2018) Therapeutic vaccines for high-risk HPV-associated diseases. Papillomavirus Res.5, 46–5810.1016/j.pvr.2017.12.00629277575PMC5887015

[5] Rodriguez‐CarunchioL., SoveralI., SteenbergenR.D.M. (2015) HPV‐negative carcinoma of the uterine cervix: a distinct type of cervical cancer with poor prognosis. BJOG122, 119–12710.1111/1471-0528.1307125229645

[6] KatkiH.A., SchiffmanM., CastleP.E. (2013) Five-year risk of CIN3+ and cervical cancer for women with HPV-positive and HPV-negative high-grade Pap results. J. Low Genit. Tract Dis.17, S50–S5510.1097/LGT.0b013e318285428223519305PMC3616447

[7] LiuD., ZhouP., ZhangL. (2011) Differential expression of Oct4 in HPV-positive and HPV-negative cervical cancer cells is not regulated by DNA methyltransferase 3A. Tumuor Biol.32, 941–95010.1007/s13277-011-0196-z21674242

[8] KwasniewskaA., PostawskiK., Gozdzicka-JozefiakA. (2011) Estrogen and progesterone receptor expression in HPV-positive and HPV-negative cervical carcinomas. Oncol. Rep.26, 153–1602149108710.3892/or.2011.1256

[9] YangG., LuX. and YuanL. (2014) LncRNA: a link between RNA and cancer. Biochim. Biophys. Acta Gene Regul. Mech.1839, 1097–110910.1016/j.bbagrm.2014.08.01225159663

[10] ZhengZ. and GaoY. (2018) Down-regulation of lncRNA snaR is correlated with postoperative distant recurrence of HPV-negative cervical squamous cell carcinoma. Biosci. Rep.13, 3810.1042/BSR20181213PMC623925630249756

[11] LuoP., JingW., ZhuM. (2017) Decreased expression of LncRNA SRA1 in hepatocellular carcinoma and its clinical significance. Cancer Biomark.18, 285–29010.3233/CBM-16030528085012PMC13020599

[12] ParkS., EomK., KimJ. (2017) MiR-9, miR-21, and miR-155 as potential biomarkers for HPV positive and negative cervical cancer. BMC Cancer17, 65810.1186/s12885-017-3642-528934937PMC5609051

[13] PengL., YuanX., JiangB. (2016) LncRNAs: key players and novel insights into cervical cancer. Tumour Biol.37, 2779–278810.1007/s13277-015-4663-926715267

[14] YangW., HongL., XuX. (2017) LncRNA GAS5 suppresses the tumorigenesis of cervical cancer by downregulating miR-196a and miR-205. Tumuor Biol.39,10.1177/101042831771131528671039

[15] ChenX., XiongD., YeL. (2019) Up-regulated lncRNA XIST contributes to progression of cervical cancer via regulating miR-140-5p and ORC1. Cancer Cell Int.19, 4510.1186/s12935-019-0744-y30858762PMC6394057

[16] LuH., HeY., LinL. (2016) Long non-coding RNA MALAT1 modulates radiosensitivity of HR-HPV+ cervical cancer via sponging miR-145. Tumuor Biol.37, 1683–169110.1007/s13277-015-3946-526311052

[17] ZhangW.Y., LiuY.J., HeY. (2019) Suppression of long noncoding RNA NCK1‐AS1 increases chemosensitivity to cisplatin in cervical cancer. J. Cell. Physiol.234, 4302–431310.1002/jcp.2719830221354

[18] YimE.K. and ParkJ.S. (2005) The role of HPV E6 and E7 oncoproteins in HPV-associated cervical carcinogenesis. Cancer Res. Treat.37, 319–32410.4143/crt.2005.37.6.31919956366PMC2785934

[19] XiaY., PadreR.C., De MendozaT.H. (2009) Phosphorylation of p53 by IκB kinase 2 promotes its degradation by β-TrCP. Proc. Natl. Acad. Sci. U.S.A.106, 2629–263410.1073/pnas.081225610619196987PMC2650315

[20] LiuY., TergaonkarV., KrishnaS. (1999) Human papillomavirus type 16 E6-enhanced susceptibility of L929 cells to tumor necrosis factor α correlates with increased accumulation of reactive oxygen species. J. Biol. Chem.274, 24819–2482710.1074/jbc.274.35.2481910455154

[21] DeyA., WongE., KuaN. (2008) Hexamethylene bisacetamide (HMBA) simultaneously targets akt and mapk pathway and represses NF-κB activity: Implications for cancer therapy. Cell Cycle7, 3759–376710.4161/cc.7.23.721319029824

[22] ChewC.L., ConosS.A., UnalB. (2018) Noncoding RNAs: master regulators of inflammatory signaling. Trends Mol. Med.24, 66–8410.1016/j.molmed.2017.11.00329246760

